# Construction of Nursing Practice Model in Case Management of Concurrent Chemotherapy and Radiochemotherapy Treatment in Cervical Cancer

This article has been retracted.

**DOI:** 10.1155/2022/5450575

**Published:** 2022-06-17

**Authors:** Liqin Tang, Yan Xing, Hui Li

**Affiliations:** Sichuan Cancer Hospital & Institute, Sichuan Cancer Center, School of Medicine, University of Electronic Science and Technology of China, Chengdu 610041, China

## Abstract

**Objective:**

To construct a case management model of synchronous radiotherapy and concurrent chemotherapy and radiochemotherapy (CRR) for cervical cancer led by nurses and carry out preliminary implementation and evaluation, so as to explore a new model of nursing practice.

**Methods:**

Totally 80 cervical cancer patients were included in this study, 43 patients were in the experimental group, and 37 patients were in the control group. The clinical data, side effects, psychological reactions, and nutritional indexes were collected before and after the intervention.

**Results:**

The results of Hospital Anxiety and Depression Scale (HADs) showed that anxiety and depression scores decreased after intervention in the experimental group, and the difference between two groups had significant after intervention (*P* < 0.05). Serum fatty acids, albumin, and cholesterol in the experimental group were decreased after the intervention. Moreover, the incidence of radiation vaginitis and radiation dermatitis had significant differences between the two groups (*P* < 0.05).

**Conclusion:**

The case management nursing practice mode of concurrent radiotherapy and chemotherapy for cervical cancer can effectively promote the self-management of risk factors, reduce the occurrence of complications, and improve the ability of self-care.

## 1. Introduction

Cervical cancer is a common gynecological tumor, which has become a serious threat to women's health. Around 500 thousand people worldwide are diagnosed with cervical cancer every year, and about 260 thousand people die. The incidence rate is gradually younger, and its annual incidence rate is increasing by about 5% [1]. It has been the world's second [2] in recent years. Concurrent radiotherapy and chemotherapy are an important treatment method for cervical cancer patients in addition to surgical treatment and have achieved good clinical results [3]. However, some patients have high tumor complexity, and there are tumor residues after the end of the concurrent radiotherapy and chemotherapy treatment cycle. This kind of tumor has a high risk of recurrence and metastasis, which undoubtedly increases the difficulty of treatment and aggravates the psychological and economic burden of patients [4].

Case management is a fully cooperative process, which includes evaluation, planning, implementation, coordination, supervision, and evaluation of selected medical services. Through full communication and a reasonable selection of available resources, it can improve service quality, reduce medical costs, and meet the health needs of patients [5]. Different disciplines have developed the definition of case management. For example, in the field of nursing, the American nurse certification center defines case management as “a flexible, systematic and cooperative method to provide and coordinate medical care services for specific people” [6]. This is a participatory process to promote the individual's choice of medical and nursing services, to meet the individual's health needs, reduce unnecessary services, reduce costs, and improve the quality and effect of nursing [7].

In the field of social work, case management is defined as a practical strategy and method of providing services. “The main goal of case management is to provide the most efficient and high-quality services for individuals with multiple needs and optimize customer service [8].” Although there are differences in definitions between different disciplines, a consensus is that case management does not stay at a certain stage or limited to a certain place but occurs in the whole process of continuous service provision, aiming to continuously meet individual needs. Case management has six core functions: evaluation, planning, contact, monitoring, publicity, and promotion [9].

A study has designed a case management program from the hospital to the community for the newly diagnosed breast cancer patients and evaluated the effect of the project on improving the quality of life and reducing medical expenses [10], and the study showed that there was no difference in medical cost between the two groups, but the uncertainty of disease in the Qianyu group decreased significantly within 6 months after diagnosis. Meanwhile, a case management model for chronic diseases was designed for patients with type 2 diabetes, and the effect of the model was tested. The results showed that after two years of case management, the clinical indicators such as HbAlc, BP, LDL, and depression and weight were improved in the intervention group, and self-management ability was higher than that in the control group [11]. However, there was no study on the case management model of synchronous radiotherapy and concurrent chemotherapy for cervical cancer.

Therefore, in our research, we construct a case management model of synchronous radiotherapy and concurrent chemotherapy for cervical cancer led by nurses and carry out preliminary implementation and evaluation, so as to explore a new model of nursing practice.

## 2. Data and Methods

### 2.1. Clinical Data

80 patients with concurrent chemoradiotherapy treatment in cervical cancer in our hospital from January 2020 to December 2022 were included in our study. This study was approved and recognized by the ethics committee of our hospital.

Inclusion and exclusion standard was as follows:

Inclusive criteria were as follows: ① primary treatment patients with radical radiotherapy and chemotherapy diagnosed with cervical cancer by pathological examination, ②postoperative radiotherapy and chemotherapy for cervical cancer, and ③ the subjects were willing to cooperate and implement the study.

Exclusion criteria were as follows: ① had a serious mental illness and ② advanced systemic tumor metastasis.

### 2.2. Method

#### 2.2.1. The Control Group (CG)

The subjects were only treated with general psychological support. The effect was evaluated after 6 months of intervention.

#### 2.2.2. The Experimental Group (EG)

On this basis, accept the case management model, as follows:

1. Preparation before nursing, establish a case management team, and the team members are the backbone of the department. Group members receive training and learning in case management mode and take up their posts after passing the examination. Provide dedicated telephones for team members. The implementers wrote their management manuals and follow-up logs to ensure complete and accurate information such as general information, surgical information, and supplementary treatment information, to compile breast cancer health education handbooks, books, videos, etc., and to screen valuable information on the network platform, and send them to patients through WeChat so that they could receive treatment intuitively. The study included 80 patients with concurrent radiotherapy and chemotherapy, all of whom signed written informed consent to the experiment
2. The implementation of the case management nursing model. ① For patients diagnosed and treated in hospital, the specialist nurse shall inform them of the purpose and implementation methods of the case management model, sign the consent after obtaining their consent, carry out nursing work for 6 months in combination with the actual clinical situation at home and abroad, and complete the evaluation, planning, implementation, feedback, and evaluation of case management using telephone follow-up, face-to-face publicity and education, SMS consultation, etc. ② The specific content of case management. Based on specialized nursing, medical staff should teach patients the method of self-care, so that they can deal with all kinds of difficult problems encountered during rehabilitation. Add WeChat and QQ numbers of patients, carry out publicity and education in various forms, provide patients with the latest scientific progress of treatment technology, and help patients build confidence; through WeChat official account and other related knowledge, improve treatment compliance. The physiological pain of cervical cancer can make patients feel low self-esteem, anxiety, and other emotions, and some patients give up themselves. Therefore, according to their family background and personality characteristics, medical staff formulate individualized psychological nursing programs and give targeted guidance
3. Personalized traditional Chinese medicine characteristic nursing. Combined with TCM syndrome differentiation, formulate corresponding food for patients. Most patients with cervical cancer have stagnation of liver qi; so, emotional nursing should be carried out one-on-one during nursing to understand the causes of their anxiety and carry out targeted intervention methods; acupoint massage, acupuncture, moxibustion, and other methods are used to help patients relieve pain

### 2.3. Data Collection

We mainly collect the general information of patients (including marital status, economic status, cultural status, and nationality: Han, Yi, and Tibetan), side effects of chemotherapy (nausea, vomiting, white blood cell number, monitoring weight gain and loss), side effects of radiotherapy (radiation proctitis, radiation cystitis, radiation vaginitis, radiation dermatitis), psychological reaction (anxiety, depression), nutritional status (albumin, prealbumin, hemoglobin), blood routine indexes before and after loading treatment, nutritional indexes, compliance with vaginal flushing, and whether the patient has lymphedema after operation.

### 2.4. Statistical Analysis

All data were analyzed by SPSS 22.0. The statistical results are expressed by mean ± standard deviation ($\bar{x}\pm s$), the data comparison is conducted by *t*-test, and the correlation analysis is conducted by person linear phase; *P* < 0.05 was the difference with statistical significance.

## 3. Results

### 3.1. Clinical Data

Totally 80 cervical cancer patients were included in this study, 43 patients were in the experimental group, and 37 patients were in the control group. Moreover, the clinical data showed that there was no significant difference in age, BMI, marital status, nation, cultural status, economic situation, and postoperative lymphedema (*P* > 0.05) (Table 1).

### 3.2. Assess the Patient's Anxiety and Depression

The results of Hospital Anxiety and Depression Scale (HADs) showed that anxiety and depression scores decreased after intervention in the experimental group, and there was significant difference between the two groups after intervention (*P* < 0.05) (Table 2 and Figure 1).

### 3.3. Nutritional Status

Serum fatty acids, albumin, and cholesterol in the experimental group were decreased after the intervention; moreover, there had a significant difference between the two groups after intervention (*P* < 0.05). However, there had no difference between the two groups in the total lymphocytes (*P* > 0.05) (Table 3).

### 3.4. Adverse Reactions

The incidence of radiation vaginitis and radiation dermatitis in the experimental group was significantly lower than in the control group, and the difference had significantly (*P* < 0.05). However, there had no difference between the two groups in the incidence of nausea, loss of weight, radiation proctitis, and radiation cystitis (*P* > 0.05) (Table 4).

## 4. Discussion

Cervical cancer is a malignant tumor that occurs in the cervix, vagina, and cervical canal. It is the most common reproductive tract cancer [12]. The incidence rate of malignant tumors is the second of gynecologic malignancies. China is one of the most frequent areas of cervical cancer. The number of new cases is about 100 thousand per year, accounting for 1/5 of the total number of new cases worldwide [13, 14].

An important feature of case management is to improve patients' health behavior and promote patients' self-management. In this study, case management nurses regularly followed up by telephone to monitor the control of risk factors of patients and correct their bad behavior in time, so as to ensure the healthy behavior of patients. The results showed that the incidence of complications of radiotherapy and chemotherapy in the experimental group was significantly lower than that in the control group. It can be seen that the case management model can effectively reduce the incidence of complications.

Due to the decline of physical function and social function, patients with cervical cancer undergoing concurrent radiotherapy and chemotherapy bear great psychological pressure and burden; so, they are more likely to accumulate negative emotions such as anxiety, depression, indifference, and inferiority complex. Such emotions not only hinder the prognosis of patients but also increase the probability of recurrence. Family members should not only bear the heavy nursing work and heavy economic burden but also face the negative emotions of patients, which is easy to produce adverse emotions such as anxiety, which will affect the nursing effect and the rehabilitation of patients.

In this study, we compared whether there were significant differences in depression and anxiety, nutrition, and adverse reactions between the experimental group and the control group. We learned that there were certain differences in depression and anxiety before and after the intervention, but the degree of depression and anxiety in the experimental group was significantly greater than that in the control group. Therefore, this study puts forward the following suggestions for the next step of case management nursing practice: ① case management nurses should pay more attention to patients' mental health and rehabilitation needs, encourage patients to express their inner feelings, and solve patients' problems in time by coordinating various relationships [15, 16]. ② In the practice of case management, case management nurses should not only teach their family members disease-related knowledge and skills but also pay attention to communication with their family members, fully understand their physical and mental needs, and provide targeted psychological and social support [17–20].

In conclusion, the case management nursing practice mode of concurrent radiotherapy and chemotherapy for cervical cancer can effectively promote the self-management of risk factors, reduce the occurrence of complications, and improve the ability of self-care.

## Figures and Tables

**Figure 1:** Hospital Anxiety and Depression Scales (HADS) were used to compare the statistical differences between the anxiety significance scores of the experimental group and the control group after intervention, so as to evaluate the level of depression and anxiety of patients. Note: compared with the experimental group, ^∗^*P* < 0.05.

**Table 1:** Comparison of clinical data between the two groups.

	Experimental group (*n* = 43)	Control group (*n* = 37)	*t*/*χ*2	*P*
Age (years)	44.05 ± 6.91	41.35 ± 7.09	3.25	0.24
BMI	17.05 ± 1.28	17.65 ± 1.06	5.29	0 .28
Smoking	17 (39.5%)	19 (51.4%)	1.96	0.69
Marital status			17.83	0.24
Married	23 (53.5%)	19 (51.4%)		
Single	6 (14%)	9 (24.3%)		
Divorced or separated	10 (23.3%)	6 (16.2%)		
Widowed	4 (9.3%)	3 (8.1%)		
Nation			3.28	0.42
Han nationality (*n*%)	32 (74.4%)	26 (70.2%)		
Yi nationality (*n*%)	10 (23.3%)	9 (24.3%)		
Zang nationality (*n*%)	1 (2.3%)	2 (5.4%)		
Cultural status			5.52	0.47
Junior high school	10 (23.3%)	3 (8.1%)		
High school/technical secondary school	13 (30.2%)	9 (24.3%)		
Junior college	13 (30.2%)	19 (51.4%)		
University and higher	7 (16.3%)	6 (16.2%)		
Economic situation			3.39	0 .35
Good	13 (30.2%)	12 (32.4%)		
Secondary	22 (51.2%)	18 (48.6%)		
Poor	8 (18.6%)	7 (18.9%)		
Postoperative lymphedema			1.35	0.39
Had	33 (76.7%)	26 (70.3%)		
No	10 (23.3%)	11 (29.7%)		

Note: compared with the control group, significant difference as *P* < 0.05.

**Table 2:** Comparison of Hospital Anxiety and Depression Scale (HADs) between the two groups after intervention (points, $\bar{x}\pm s$).

	Time	Experimental group (*n* = 43)	Control group (*n* = 37)	*t*	*P*
Anxiety	Before intervention	10.37 ± 2.10	10.19 ± 2.01	0.52	0.096
	After intervention	5.63 ± 2.35	9.09 ± 2.42	5.78	<0.001
	*t*	24.9	5.78	—	—
	*P*	<0.001	0.02	—	—

Depression	Before intervention	10.67 ± 2.37	10.31 ± 2.09	0.54	0.27
	After intervention	6.31 ± 2.89	9.39 ± 2.32	6.32	<0.001
	*t*	16.91	7.15	—	—
	*P*	<0.001	<0.001	—	—

Note: compared with the control group, significant difference as *P* < 0.05.

**Table 3:** Comparison of nutritional status between the two groups before and after intervention (points, $\bar{x}\pm s$).

	Time	Experimental group (*n* = 43)	Control group (*n* = 37)	*t*	*P*
Serum fatty acids	Before intervention	1.33 ± 0.10	1.19 ± 0.32	1.52	0.086
	After intervention	0.63 ± 0.35	1.09 ± 0.42	5.78	<0.001
	*t*	3.29	2.18	—	—
	*P*	0.042	0.062	—	—

Serum albumin	Before intervention	43.67 ± 4.37	44.32 ± 2.49	0.54	0.37
	After intervention	36.32 ± 1.99	47.29 ± 2.12	16.42	0.0001
	*t*	8.91	7.15	—	—
	*P*	0.0001	0.321	—	—

Total lymphocytes	Before intervention	1.67 ± 0.37	1.42 ± 0.09	2.34	0.39
	After intervention	1.01 ± 2.89	1.39 ± 2.32	1.32	0.056
	*t*	3.91	7.15	—	—
	*P*	0.053	0.076	—	—

Serum cholesterol	Before intervention	170.65 ± 12.37	178.31 ± 20.09	0.54	0.27
	After intervention	106.31 ± 3.19	169.39 ± 2.29	6.32	0.0002
	*t*	14.31	3.15	—	—
	*P*	0.0003	0.045	—	—

Note: compared with the control group, significant difference as *P* < 0.001.

**Table 4:** Comparison of adverse reactions between two groups.

Group	Nausea	Lose weight	Radiation vaginitis	Radiation dermatitis	Radiation proctitis	Radiation cystitis
Experimental group	7 (16.3%)	8 (18.6%)	9 (20.9%)	9 (20.9%)	14 (32.6%)	5 (11.6%)
Control group	10 (27%)	7 (18.9%)	15 (40.5%)	16 (43.2%)	11 (29.7%)	7 (18.9%)
*t*	7.153	3.621	6.378	6.378	4.061	9.737
*P*	0.643	0.742	0.034	0.038	0.081	0.382

Note: compared with the control group, significant difference as *P* < 0.05.

## Data Availability

The data used to support this study is available from the corresponding author upon request.
